The article "Water Treatment Using Natural Coagulant and Electrocoagulation Process: A Comparison Study" was published in 2022. Journal: Int J Anal Chem.

# Water Treatment Using Natural Coagulant and Electrocoagulation Process: A Comparison Study

**DOI:** 10.1155/2022/4640927

**Published:** 2022-09-29

**Authors:** Tofik Gali Aba Lulesa, Dejene Beyene, Million Ebba, Goshu Kenea

**Affiliations:** ^1^Department of Water Supply and Environmental Engineering, Faculty of Civil and Environmental Engineering, Jimma Institute of Technology, Jimma University, P.O. Box-378, Jimma, Ethiopia; ^2^Department of Civil Engineering, Faculty of Civil and Environmental Engineering, Jimma Institute of Technology, Jimma University, P.O. Box-378, Jimma, Ethiopia

## Abstract

Water treatment is the primary consideration before utilizing water for different purposes. Surface water is highly vulnerable to pollution, either due to natural or anthropogenic processes. The main targets of this study were to investigate surface water treatment using *Moringa Oleifera* (MO), the electrocoagulation process (EC), and the *Moringa Oleifera* assisted electrocoagulation process (MOAEC). The *Moringa Oleifera*, EC process, and *Moringa Oleifera*-assisted EC process are effective mechanisms for the removal of COD (Chemical Oxygen Demand), BOD (Biological Oxygen Demand), TDS (Total Dissolved Solids), phosphate, TSS (Total Suspended Solids), and color from surface water. Different operating parameters such as pH (5–11), the dosage of coagulant (0.2–0.5 g), contact time or reaction time (20–50 minutes), current (0.2–0.5 A), and settling time (5–20 minutes) were considered. The maximum removal efficiency using *Moringa Oleifera* and the EC process was COD (85.48%), BOD (78.50%), TDS (84.5%), phosphate (95.70%), TSS (93.90%), color (94.50%), and COD (90.50%), BOD (87%), TDS (97.50%), phosphate (89.10%), TSS (95.80%), and color (96.15%), respectively. Similarly, with the application of MOAEC, 91.47%, 89.35%, 97.0%, 90.20%, 9.10%, and 95.70% of COD, BOD, TDS, phosphate, TSS, and color were removed, respectively. The EC process and MOAEC were more effective in the removal of COD, BOD, TDS, TSS, and color than using MO. More phosphate was removed using MO than the EC process and MOAEC. Additionally, the effects of different operating parameters were studied on the removal efficiency.

## 1. Introduction

As a human being in this global village, “water” is one of the most important needs [1, 2], and for all living things and activities, as well as for preserving the environment and its resources, water is vitally important [3–5]. Most of Earth's surface is covered by water, which covers more than two-thirds of the planet's surface, but most of it is salty and useless [6]. In addition to this, the world's water resources could also be contaminated due to a variety of natural and man-made factors [7, 8]. Urbanization [9–12], industrialization [10, 11, 13, 14], agricultural, [13–15] surface runoff, and sediment transport [2] are some of the factors considered in the deterioration of the parameters of water quality.

On a global scale, at least four billion people do not have access to clean drinking water, or they believe that it is unsafe to drink [16]. World, continent, and country-level human health are directly affected by drinking water quality [17]. Many countries, especially those in developing countries, have poor water quality, which has led to several waterborne diseases [4, 11, 18, 19].

Diverse water treatment technologies have been created in response to the alarming condition of water shortages to assure the creation of an appropriate water supply and quality to fulfill the demand and preserve the availability of clean water resources. These technologies can generally be divided into three groups: physical, chemical, and biological processes [20]. Without significantly altering the chemical or biological properties of the treated water, physical treatment unit operations solely rely on the physical separation of contaminants from water/wastewater [21]. Chemical treatments are known as additive procedures because additional chemicals are needed for them to interact with the intended pollutants and remove them, and the fundamental objective of biological unit procedures, which use microorganisms for the biodegradation of pollutants in water/wastewater, is to lower the organic content and nutrients in the water/wastewater [21].

Whatever type of water treatment process is used, it must be considered in a variety of situations, including the effectiveness of the technology, ease of implementation, environmental friendliness, cost-effectiveness, and skilled manpower required to run the technology.

Electrocoagulation (EC) is an electrochemical process for water and wastewater treatment that is based on electrochemically dissolving cationic metallic species in situ by oxidizing a sacrificial anode only with the application of electric current [22]. By using electrical energy to dissolve the metals from the electrode surface and destabilize colloidal suspensions, electrocoagulation causes pollutants to flocculate and float [23]. In comparison to traditional treatment methods, the electrocoagulation (EC) process is a promising and fairly environmentally friendly technology for the removal of contaminants from water and wastewater due to its ease of installation and operation; no need for chemical addition; relatively low operation; and maintenance cost; low sludge production; and high removal efficiency of pollutants [24]. Some studies were conducted on water treatment utilizing the electrocoagulation process under different operating parameters for the removal of arsenic [25, 26], fluoride [25], bromide [27, 28], sulfate [29], chromium [30], copper [31], and selenium [32].

Metal-based coagulants are the most often used chemical to support the flocculation-coagulation processes in the treatment of water and wastewater and they function admirably in the treatment of numerous water and wastewater kinds with distinct properties [33]. However, to attain green technology and sustainable processes, some researchers suggest using plant-based coagulants as an alternative to the widely used metal-based coagulant [34–38].

Natural coagulants used for water and wastewater treatment have numerous advantages [39], such as being eco-friendly; the flocculation technique is more cost-effective and efficient; it is a cheap and simple approach for developing nations; it does not affect water taste; it does not cause health problems; and the small amount of sludge that is precipitated is biodegradable and safe for human health and the environment.

*Moringa oleifera* is a type of natural coagulant used for the treatment of water and wastewater. An investigation was conducted into the water and wastewater treatment for the elimination of color, COD, BOD, dissolved oxygen, TSS, TDS, and turbidity [36, 39, 40]. In this study, the application of electrocoagulation and *Moringa Oleifera* on surface water treatment for the removal of color, TDS (Total Dissolved Solids), COD (Chemical Oxygen Demand), BOD (Biological Oxygen Demand), and phosphate was discussed separately.

Additionally, the removal efficiency of color, TDS (Total Dissolved Solids), COD (Chemical Oxygen Demand), BOD (Biological Oxygen Demand), and phosphate using *Moringa Oleifera* assisted electrocoagulation was studied. Furthermore, different factors that influence the removal efficiency of color, TDS (Total Dissolved Solids), COD (Chemical Oxygen Demand), BOD (Biological Oxygen Demand), and phosphate were discussed.

## 2. Materials and Methods

### 2.1. Materials

Surface water supply was collected from the Awetu River, Jimma Zone, and Oromia Regional State, Ethiopia. Surface water was collected using the grab sampling technique for sampling, and was then kept in a refrigerator (4°C) to prevent changes in the quality of water. The materials used for this study were a beaker, magnetic stirrer (model RHB2), desiccator, drying oven, filter paper, COD reactor (Hatch 45600-02), COD digester, COD kit, BOD incubator, DO meter, electrode (Al-Al), DC-power supply (WYJ-o-15 V/5 A), spectrophotometer (model 6700), vacuum pump, vacuum hood, heaters, conical flasks, pH meter, standard flasks, Erlenmeyer flasks, measuring cylinder, plastic bottles, burettes, thermometer, funnel, suction flask, wash bottle, porcelain dish, weighing balance (model Pw-124), weighing balance (model Pw-124), filtration apparatus, graduated cylinder, turbidity meter (Wag-WT3020), pH meter (pH 3310), and ultraviolet (UV) lamp (model PUV-1022).

### 2.2. Methods

#### 2.2.1. Experimental Procedure for Electrocoagulation Process

An experimental investigation was conducted at standard room pressure and temperature. As shown in Figure 1, an electrocoagulation process was used in a 1-liter glass beaker as an electrocoagulation cell. An aluminum electrode was used that has a dimension of 6 cm, 13 cm, and 0.2 cm for length, width, and thickness respectively. An effective surface area of the electrode was adjusted to 55 cm^2^ throughout the experiments.

Once the water sample was added to the electrocoagulation cell, the EC cell was placed on a magnetic stirrer. A magnetic stirrer bar also placed inside the EC contains water samples that mix water samples based on the seed of the magnetic stirrer. An aluminum electrode was connected to an anode and cathode and then inserted into the electrocoagulation cell containing the water sample. The distance between electrodes was adjusted to 2 cm. Then, electrodes from the anode and cathode are connected to a DC-power supply with electrical wires. By adjusting all operating parameters (reaction time, pH, and current), the removal percentages of color, turbidity, TDS, COD, and phosphate were evaluated.

#### 2.2.2. Experimental Procedure Using *Moringa Oleifera*

*Moringa Oleifera* seed powder was collected from a locally available market and its powder preparation was based on an experimental procedure. *Moringa Oleifera* seeds are first dried with sunlight to remove the moisture content. Mortar, pan, sieve, paper, and oven-dry were the instruments used for the preparation of *Moringa Oleifera* seed powder. Once the husks were removed from the *Moringa Oleifera* seeds, they were placed in a mortar and crushed, and then they were placed in an oven to dry with the using pan at 105°C for 7 hours [36]. Then, using a jar test, different water characteristics (% color, % turbidity, % TDS, % COD, and % phosphate) were evaluated after adjusting the dosage of *Moringa Oleifera* seed powder, pH, settling time, and contact time as shown in Figure 2.

#### 2.2.3. Experimental Procedure of *Moringa Oleifera* Assisted EC Process

One of the practical methods for expanding the use and proving the efficacy of natural coagulants is to combine them with other treatment technologies, much like how traditional inorganic coagulants are combined with other processes. A relatively novel method for enhancing the overall performance of an integrated system is the use of natural coagulant (*Moringa Oleifera* seed) in conjunction with the EC process.

Some research was conducted in keeping one factor and evaluating the removal of different parameters from water, and investigating the effects of each factor separately [22, 36, 41] However, in this study, based on the adjusted values of factors either for the electrocoagulation process or Moringa Oleifera an experiment was conducted just uniformly with the increase of each factor without keeping one factor constant.

*Moringa Oleifera*-assisted EC process was performed similarly to the EC process as shown in Figure 1. But a different dosage of *Moringa Oleifera* seed powder (0.2, 0.3, 0.4, and 0.5 g) was added to the EC setup shown in Figure 1.

### 2.3. Analysis

Different empirical formulas were used for the analysis of surface water characteristics based on the initial and final concentrations of pollutants. The removal efficiencies of color [22], phosphate [42], TDS [43], COD [36, 44], and BOD [44] were calculated using equations ((1)–(5)).

(1) $$\begin{array}{c} \%\text{Color Removal}=\;\frac{{\text{Abs}}_{i}-{\text{Abs}}_{f}}{{\text{Abs}}_{i}}*100, \end{array}$$

where, Abs_*i*_ and Abs_*f*_ are initial and final absorbance.

(2) $$\begin{array}{c} \%\text{Phosphate Removal}=\;\frac{C_{i}-C_{t}}{C_{i}}*100, \end{array}$$

where, *C*_*i*_ and *C*_*t*_ are initial and final phosphate registered at different times.

(3) $$\begin{array}{c} \%\text{TDS Removal}=\;\frac{C_{o}-C_{f}}{C_{o}}*100, \end{array}$$

where, *C*_*o*_ and *C*_*f*_ are initial and final concentration of TDS respectively.

(4) $$\begin{array}{c} \%\text{COD Removal}=\;\frac{{\text{COD}}_{i}-{\text{COD}}_{f}}{{\text{COD}}_{i}}*100, \end{array}$$

where, COD_*i*_ and COD_*f*_ are initial and final concentration of COD.

(5) $$\begin{array}{c} \%\text{BOD Removal}=\;\frac{{\text{BOD}}_{i}-{\text{BOD}}_{f}}{{\text{BOD}}_{i}}*100, \end{array}$$

where, BOD_*i*_ and BOD_*f*_ are the initial and final BOD measured at different time.

## 3. Results and Discussion

### 3.1. Removal Efficiency COD, BOD, TDS, Phosphate, TSS, and Color

The removal efficiency was evaluated for COD, BOD, TDS, phosphate, TSS, and color from water using *Moringa Oleifera* as a coagulant, electrocoagulation process, and *Moringa Oleifera*-assisted electrocoagulation process. While using *Moringa Oleifera* seed powder, coagulant dosage (0.2, 0.3, 0.4, and 0.5 g), pH (5, 7, 9, and 11), contact time (20, 30, 40, and 50 minutes) and settling time (5, 10, 15, and 20 minutes) are considered as operating parameters on the removal efficiency. During the electrocoagulation process, the pH of surface water and contact time or reaction time is fixed to be the same as in the treatment process using the *Moringa Oleifera* process. However, the electric current applied was adjusted to 0.2, 0.3, 0.4, and 0.5 A.

At pH 5, the removal efficiency of COD (78.30%), BOD (70%), TDS (81.20%), phosphate (85%), TSS (87.50%), color (89%), and COD (80%), BOD (81%), TDS (94.20%), phosphate (81.20%), TSS (87%), and color (92.80%) using *Moringa Oleifera* and electrocoagulation processes, respectively. In this case, the dosage of *Moringa Oleifera* was 0.2 g at 20 minutes of contact time and 5 minutes of settling time. But the removal efficiency was achieved at 20 minutes of reaction time and 0.2 A of current with the electrocoagulation process. The removal percentages of TSS and phosphate were higher using *Moringa Oleifera* than in the electrocoagulation process, but the removal efficiency of COD, BOD, TDS, and color using electrocoagulation was higher than using *Moringa Oleifera* as a coagulant at pH 5.

Increasing the pH to 7 results in the increasing removal efficiency of COD, BOD, TDS, phosphate, TSS, and color using both the *Moringa Oleifera* and electrocoagulation processes. The removal percentages of COD (79.20%), BOD (74.30%), TDS (83.10%), phosphate (89.50%), TSS (91%), and color (92.70%) were removed with a dosage of 0.3 g of *Moringa Oleifera* at 30 minutes of contact time and 10 minutes of settling time. Similarly, using the EC process, when the reaction time was 30 minutes and the current applied was 0.3 A, the removal efficiency of COD, BOD, TDS, phosphate, TSS, and color were 87.30%, 83.10%, 83.10%, and 95.70%, 84.90%, 90.90%, and 94.50%, respectively. So, at pH 7, the higher removal efficiency was achieved for phosphate and TSS using *Moringa Oleifera*, and more COD, BOD, TDS, and color were also removed using the EC process.

When pH was 9, the removal efficiency of pollutants was increased, similar to at pH 5 and 7. The removal percentages of COD, BOD, TDS, phosphate, TSS, and color were increased to 81.89%, 76.90%, 83.52%, 93.28%, 92.50%, and 93%, respectively, using *Moringa Oleifera*. Similarly, with the application of the electrocoagulation process, the better removal efficiency was achieved for COD (89%), BOD (85.70%), TDS (93.50%), TSS (96.40%), and color (95.78%) compared to using *Moringa Oleifera*. However, in the case of phosphate removal, using *Moringa Oleifera* was better than utilizing the electrocoagulation process.

Another experiment was also conducted at pH 11 using *Moringa Oleifera* and the EC process. In both cases, good removal percentages of COD, BOD, TDS, phosphate, TSS, and color were achieved with the consideration of influencing parameters. Using *Moringa Oleifera* seed powder of 0.5 g, 50 minutes of contact time, and 20 minutes of settling time, 95.70% of phosphate and 94.50% of color were removed from surface water. The removal percentages for COD, BOD, TDS, and TSS were also good, even if they were not enough compared to using the EC process. Applying the EC process at pH 11, by increasing the current to 0.5 A and reaction time to 50 minutes, maximum removal efficiency of COD (90.50%), BOD (87%), TDS (97.50%), TSS (95.80%), and color (96.15%) compared to using *Moringa Oleifera* for COD (85.48%), BOD (78.50%), TDS (84.50%), TSS (93.90%), and color (94.50%).

*Moringa Oleifera* was found to have a high percentage of phosphate removed compared to the EC process at different influencing parameters. Similarly, at pH, 5, 7, 9, and 11, the EC process was effective in the removal of COD, BOD, TDS, and color relative to *Moringa Oleifera* seed powder.

Additional experiments were also conducted on the removal degree of COD, BOD, TDS, phosphate, TDS, and color from surface water using the *Moringa Oleifera* enhanced electrocoagulation process. The investigation was conducted at pH (5, 7, 9, and 11), current (0.2, 0.3, 0.4, and 0.5 A), the dosage of *Moringa Oleifera* (0.2, 0.3, 0.4, and 0.5 g), and reaction time of (20, 30, 40, and 50 minutes). Any water sample that contains more electric conductivity that undergoes an electrocoagulation process and better removal efficiency is enhanced. Sometimes, when water sample electric conductivity was lower, different types ofsupporting electrolytic such as Na_2_SO_4_, KCl, NaCl, and NaHCO_3_ will be added to achieve better removal efficiency [45]. To increase electrolytic conductivity and prevent the formation of an oxide layer, minimize the ohmic drop, and therefore increase power density, a supportive electrolyte is added [45]. Regarding the relationship between pH and electrical conductivity, Electrical conductivity is a nonspecific measurement of the concentration of both positively and negatively charged ions in a sample, whereas pH measures a particular hydrogen ion. Hence, water contains more ions, indicating higher electrical conductivity, whether it may be in acidic or basic conditions. In this study, the electrical conductivity of water was not measured, and it directly focused on the pH, current, and *Moringa Oleifera* powder.

When pH was 5, 7, 9, and 11, the removal percentages of COD were 83.50%, 86.50%, 87.90%, and 91.47% at 0.2, 0.3, 0.4, and 0.5 A, respectively. This was achieved at reaction times of electrocoagulation processes of 20, 30, 40, and 50 minutes. In this case, the removal of COD is better than using the *Moringa Oleifera* assisted EC process than using the EC process and *Moringa Oleifera*.

Similarly, the removal percentage of BOD was 79.50%, 82.90%, 85.20%, and 89.35% at pH 5, 7, 9, and 11, respectively. These results were achieved at reaction times of 20, 30, 40, and 50 minutes and with 02, 0.3, 04, and 0.5 A of current. When the pH was 11, the current was 0.5 A, the dosage of *Moringa Oleifera* was 0.5 g, and the reaction time was 50 minutes. *Moringa Oleifera* assisted EC process removed COD, BOD, TDS, phosphate, TSS, and color up to 91.47%, 89.35%, 97.60%, 90.20%, 96.10%, and 95.70%, respectively.

In terms of general removal degree, the *Moringa Oleifera*-assisted EC process removes a higher percentage of COD, BOD, and TSS than the EC process and *Moringa Oleifera* alone. However, the highest removal percentages of phosphate were obtained using *Moringa Oleifera*, as well as for TDS and color, utilizing the EC process.

Generally, the application of *Moringa Oleifera*, electrocoagulation process, and *Moringa Oleifera* assisted EC process was effective for the removal of pollutants from surface water with consideration of different influencing parameters.

### 3.2. Influences of Operating Parameters

#### 3.2.1. Effects of pH

The major operating parameter in water treatment using *Moringa Oleifera* and the EC process is pH. The pH of the water was adjusted to 5, 7, 9, and 11 using NaOH and H_2_SO_4_. Increasing pH, using *Moringa Oleifera*, resulted in the increasing removal efficiency of COD, BOD, TDS, phosphate, TSS, and color. The concentration of hydrogen ions can have an impact on the effectiveness of pollutant removal (pH level). The higher removal percentage of pollutants is related to the high generation of hydrogen ions in water under acidic, neutral, or basic conditions. So, by increasing the pH of water from 5 to 11, the removal percentage of COD, BOD, TDS, phosphate, TSS, and color increases using *Moringa Oleifera*. However, according to [36], increasing the pH to 9 increased the removal efficiency of pollutants, and further increasing the pH resulted in the reduction of pollutants. Similarly, while using the EC process and *Moringa Oleifera*, the removal efficiency of COD, BOD, TDS, phosphate, TSS, and color was increased as pH increased from 5 to 7, from 7 to 9, and then from 9 to 11. Figures 3(a) and 3(b) show the removal efficiency of COD and BOD using *Moringa Oleifera* (MO), electrocoagulation process (EC), and *Moringa Oleifera* assisted electrocoagulation process (MOAEC) increases as pH increases, respectively. This is due to the creation of hydrogen gas and the accumulation of hydroxide following the reduction of water in the cathode [46].

#### 3.2.2. Effects of Dosage

The quantity of *Moringa Oleifera* powder added was also another factor affecting the removal of pollutants from water. In this study, the dosage of *Moringa Oleifera* powder was fixed at 0.2, 0.3, 0.4, and 0.5 g as shown in Figure 4. Using only *Moringa Oleifera*, the removal efficiency of COD, BOD, TDS, phosphate, TSS, and color was increased as the dosage was increased. Similarly, the removal percentages of COD, BOD, TDS, phosphate, TSS, and color were increased as the dosage of *Moringa Oleifera* was increased from 0.2 to 0.3 g, 0.3 to 0.4 g, and from 0.4 to 0.5 g using *Moringa Oleifera* assisted electrocoagulation as shown in Figure 4. As illustrated in Figures 4(a) and 4(b), the removal percentages of TDS, and TSS, and the removal percentages of phosphate and color increase as the dosage of *Moringa Oleifera* increases respectively. The removal efficiency of the pollutants was increased by increasing the *Moringa Oleifera* dosage until an optimum dosage was required [47]. Increased dosages of *Moringa Oleifera*, over and above what is necessary for best results, may be obtained because of the saturation of the polymer bridge site since *Moringa Oleifera* seeds are known to have a cationic character [47]. This may be caused by the reversal of a charge that resulted in the rise of residual turbidity as a result of the destabilized particles being restored to their original state [47].

#### 3.2.3. Effects of Contact Time

The major factor influencing water treatment using *Moringa Oleifera* is contact time. It is a time when a coagulant reacts with a pollutant once it is added to water using the jar test. It is also considered as reaction time in the case of an electrocoagulation process. The investigation was conducted by adjusting the contact time or reaction time to 20, 30, 40, and 50 minutes for *Moringa Oleifera* using a jar test and *Moringa Oleifera* assisted electrocoagulation process as shown in Figure 5. The removal efficiency of COD, BOD, TDS, phosphate, TSS, and color was good at lower reaction times or contact times (20 and 30 minutes), and by increasing the contact or reaction time to 40 minutes, the removal efficiency achieved was greater than the lower election time in both the *Moringa Oleifera* using jar test and the *Moringa Oleifera*-assisted EC process, as shown in Figure 3. As shown in Figures 5(a) and 5(b), the removal efficiency of TSS and color increased as the reaction or contact time increased, respectively. Further increasing the reaction time or contact time to 50 minutes, a higher removal degree of COD, BOD, TDS, phosphate, TSS, and color was achieved. This is due to the probability of the particle formed reacting with a pollutant while the contact time is increased.

#### 3.2.4. Effects of Settling Time

After the coagulation-flocculation process takes place using the jar test, the sample of water must be settled to evaluate the removal efficiency of COD, BOD, TDs, phosphate, TSS, and color. The settling time was adjusted to 5, 10, 15, and 20 minutes as shown in Figure 6. After 5 minutes of settling time, the removal of those parameters was good, and by increasing the settling time to 10 minutes, the removal efficiency was increased, as shown in Figure 6. Further increasing the settling time to 15 minutes, and then, to 20 minutes, the removal efficiency of COD, BOD, TDS, phosphate, TSS, and color was increased. Increasing the settling time increased the removal of% COD, % BOD, and% TDS (Figure 6(a)) and% phosphate, % TSS, and% color (Figure 6(b)). The increase in settling time results in the increase of pollutants from the water. This may be due to the *Moringa Oleifera* (coagulant) attracting the pollutants in the water and settling at the bottom of the testing beaker while increasing the settling time.

#### 3.2.5. Effects of Current

Current is a major factor in the electrocoagulation process that refers to the amount of electric current applied in amperes to an electrocoagulation cell or reactor. The driving force behind electrochemical reactions is the applied electric current that pertains to the oxygen discharge at the anode and the development of hydrogen at the cathode [48]. In this study, the current for the EC process was fixed to 0.2, 0.3, 0.4, and 0.5 A to evaluate the removal efficacy of COD, BOD, TDS, phosphate, TSS, and color with the combination of other operating parameters as shown in Figure 7. The removal efficiency changes when the amount of electric current used during the electrocoagulation process is altered. When 0.2 and 0.3 A were applied to the EC reactor, the removal percentages of COD, BOD, TDS, phosphate, TSS, and color achieved were good. By increasing the current to 0.4 A, more removal efficiency was achieved than at 0.2 and 0.3 A. While further current was applied, more removal percentages were achieved. Figures 7(a)–7(c), illustrate, that the removal efficiency of COD, BOD, TDS, phosphate, TSS, and color were increased as the current was increased. The production of hydroxide flocs and bubble density increased when the current values were raised, accelerating the removal of contaminants from water or wastewater [49].

The good removal of contaminants from the water was achieved while the electric current was a progressive increase [22]. This can be observed that the rate of coagulant and bubble generation is determined by the applied current, and this can improve the effectiveness of pollutant removal [22].

## 4. Conclusions

Water treatment is a crucial task needed before a water supply for different purposes. The treatment technology and process must be effective while being selected from different perspectives. *Moringa Oleifera* seed is a natural coagulant that is used for the treatment of water and has numerous advantages relative to synthetic coagulants. Followed by the coagulation-flocculation process, *Moringa Oleifera* seed powder can remove pollutants from surface water. Dosage of *Moringa Oleifera* seed powder, pH, contact time, and settling time are the main factors considered to evaluate the removal of COD (Chemical Oxygen Demand), BOD (Biological Oxygen Demand), TDS (Total Dissolved Solids), phosphate, TSS (Total Suspended Solids), and color, and the study showed that it was an effective process. Similarly, the EC process is also another simple technology for the treatment of water only with the application of electric current using sacrificial electrodes. With an electric current applied, pH, and reaction time as operating parameters, the EC process was effective in the elimination of COD, BOD, TDS, phosphate, TSS, and color from surface water.

Additionally, the *Moringa Oleifera*-assisted electrocoagulation (MOAEC) process is performed by the addition of *Moringa Oleifera* seed powder to the EC process. The study showed that the MOAEC process is effective in the removal efficiency of COD, BOD, TDS, phosphate, TSS, and color from surface water. Generally, *Moringa Oleifera* (MO), the electrocoagulation process (EC), and the *Moringa Oleifera*-assisted electrocoagulation process were all found to be effective methods for removing color, TSS, TDS, BOD, COD, and phosphate from surface water.

## Figures and Tables

**Figure 1:** Electrocoagulation process experimental setup.

**Figure 2:** Jar test.

**Figure 3:** Effects of pH on COD (a) and BOD (b) removal efficiency using *Moringa Oleifera* (MO), electrocoagulation (EC), and *Moringa Oleifera*-assisted EC (MOAEC).

**Figure 4:** Effects of dosage on TDS and TSS removal efficiency (a) and phosphate and color removal efficiency (b) using *Moringa Oleifera* (MO) and *Moringa Oleifera*-assisted EC process (MOAEC).

**Figure 5:** Effects of time on removal efficiency of TSS (a) and color (b) using *Moringa Oleifera* (MO), the electrocoagulation process (EC), and the *Moringa Oleifera*-assisted EC process (MOAEC).

**Figure 6:** Effects of settling time on COD, BOD, and TDS removal efficiency (a) and phosphate, TSS, and color removal efficiency (b) using *Moringa Oleifera* (MO).

**Figure 7:** Effects of current on COD and BOD removal efficiency (a), TDS and TSS removal efficiency (b), and phosphate and color removal efficiency (c) using EC process and *Moringa Oleifera*-assisted EC process (MOAEC).

## Data Availability

The data used to support the findings of this study are available from the corresponding author upon request.
